The article "Utilization of Pectin from Okra as Binding Agent in Immediate Release Tablets" was published in 2021. Journal: Biomed Res Int.

# Utilization of Pectin from Okra as Binding Agent in Immediate Release Tablets

**DOI:** 10.1155/2021/6002286

**Published:** 2021-11-30

**Authors:** Frederick W. A. Owusu, Mariam E. Boakye-Gyasi, Philomena Entsie, Marcel T. Bayor, Kwabena Ofori-Kwakye

**Affiliations:** ^1^Department of Pharmaceutics, Faculty of Pharmacy and Pharmaceutical Sciences, Kwame Nkrumah University of Science and Technology, Kumasi, Ghana; ^2^Department of Herbal Medicine, Faculty of Pharmacy and Pharmaceutical Sciences, Kwame Nkrumah University of Science and Technology, Kumasi, Ghana

## Abstract

Polymeric materials from plants continue to be of interest to pharmaceutical scientists as potential binders in immediate release tablets due to availability, sustainability, and constant supply to feed local pharmaceutical industries. Paracetamol tablet formulations were utilized in investigating the potential binding characteristics of pectin harnessed from various okra genotypes (PC1-PC5) in Ghana. The pectin yields from the different genotypes ranged from 6.12 to 18.84%w/w. The pH of extracted pectin ranged from 6.39 to 6.92, and it had good swelling indices and a low moisture content. Pectin extracted from all genotypes were evaluated as binders (10, 15, and 20%w/v) and compared to tragacanth BP. All formulated tablets (F1-F18) passed the weight uniformity, drug content, hardness, and friability tests. Based on their crushing strength, tablets prepared with pectin from the various genotypes were relatively harder (*P* ≤ 0.05) than tablets prepared with tragacanth BP. Tablets prepared with pectins as binders at 10%w/v and 15%w/v passed the disintegration and dissolution tests with the exception of PC4 at 15%w/v. Incorporation of pectin from all genotypes (excluding PC5) as a binder at concentrations above 15%w/v (F13, F16, F14, and F15) produced tablets which failed the disintegration test and showed poor dissolution profiles. Thus, pectin from these genotypes can be industrially commodified as binders in immediate release tablets using varying concentrations.

## 1. Introduction

Binders are pharmaceutical excipients which are polymeric in nature and possess cohesive as well as adhesive properties. The mode of incorporation of the binding agent has an effect on formulated tablet characteristics such as hardness, friability, and tensile strength. They are added to the granule mix to improve agglomerate formation, granule flowability, and compressibility [1, 2].

Owing to their numerous pharmaceutical applications such as diluents, binders, disintegrant in tablets, and thickeners in liquid dosage forms, plant-derived polymers have gained considerable interest in recent years. Such polymers are biocompatible, inexpensive, readily available, and are superior to synthetic pharmaceutical additives due to low cost, low toxicity, and nonirritant nature. This enables them to compete with the current commercially produced synthetic excipients [3, 4]. Plant-based polymers such as gums and mucilage have been researched for their use as binders in immediate release tablets due to their reported advantages over synthetic polymers as binders [5–7]. However, pectin is another potential natural source for a binder that has received less attention.

The article "Utilization of Pectin from Okra as Binding Agent in Immediate Release Tablets" was published in 2021. Journal: Biomed Res Int.

Pectin is a complex mixture of polysaccharides (mainly D-galacturonic acid (GalA) units, joined in chains by means of a-(1-4) glycosidic linkage) in higher plants. Pectin concentrations are greatest in the middle lamella of the cell wall, gradually decreasing as one approaches the plasma membrane. It has been used effectively as a thickening agent and a colloidal stabilizer in the food and beverage sector for many years [3, 8]. Even though pectin from citrus and mango peel have been investigated as potential binding agents in immediate release tablets, these two major sources of pectin have long maturity periods [9–11]. This makes the use of their pectin in the pharmaceutical industry as an excipient unpopular. In order to overcome these challenges, alternative sources of pectin being investigated include sugar beet waste from sugar manufacturing, sunflower heads, and recently cocoa and okra pods which have relatively shorter plant maturity periods [11, 12].

Several species of okra are cultivated in different parts of the world mainly as food and for economic reasons. Their very short maturation period and potential for producing significant quantities of pectin for medicinal application is an attractive niche for pharmaceutical researchers to investigate [13, 14]. Despite the fact that pectin has been isolated from okra and studied as a drug release modifier, currently, there is limited information on the binding properties of okra pectin and the effect of genotypic variations on the potential of okra pectin as a binder [15, 16]. This study sought to research into the potential and comparative binding properties of pectin from five (5) okra genotypes in Ghana. Investigating the binding characteristics of okra pectin from various genotypes will offer the essential knowledge on okra pectin's potential as a binder and the influence of genotypes on okra pectin's binder quality. This study will ultimately assess the possibility for commercialization of okra grown in Ghana as a binder in immediate release tablets.

## 2. Materials and Methods

### 2.1. Materials

Okra (Abelmoschus esculentus L.) genotypes: PC1 (Penkruma), PC2 (Agbagoma), PC3 (Asha), PC4 (Sengavi), and PC5 (Balabi) were obtained from various markets in Ghana and authenticated at the Department of Horticulture, KNUST, Ghana. Maize starch BP was from UK Chemicals. Paracetamol BP was from Biotech Co., China. Tragacanth BP was from Sigma-Aldrich. Talc and lactose were from BDH Laboratory Chemicals Poole, UK.

The article "Utilization of Pectin from Okra as Binding Agent in Immediate Release Tablets" was published in 2021. Journal: Biomed Res Int.

### 2.2. Methodology

#### 2.2.1. Extraction of Pectin

Pectin was extracted and isolated as described by [15, 17]. The okra pods were cut open, and the seeds removed. The separated okra pods were sun dried and milled to powder. The dried okra powder (20 g) was defatted with petroleum ether (1 g : 10 mL) for 4 hours. Aqueous extraction of defatted okra powder with 0.1 M phosphate buffer (1 g powder : 30 mL buffer solution), pH 6.0, at 80°C was carried out for 1 hour. Centrifugation was used to isolate the soluble polymer from the insoluble residue after extraction (3000 rpm for 10 min at 25°C). Evaporation at 80°C concentrated the solubilized pectin in the supernatant, which was then precipitated with 96% (v/v) aqueous ethanol. After the ethanol extraction, the samples were washed in isopropanol and then freeze dried. The freeze dried pectins were stored in air tight containers in desiccators to prevent absorption of moisture pending further analysis.

#### 2.2.2. Physicochemical Properties of Extracted Pectin

We followed the methods of [18] in determining the swelling index and water holding capacity of the extracted pectins. One (1) gram of pectin from each genotype was weighed into a 10 ml measuring cylinder, and the initial volume (Vi) was noted. Distilled water was added to the 10 ml mark. The measuring cylinder was stoppered, mixed lightly, and allowed to stand for 24 hours. The volume occupied by the pectin after 24 hours was also noted (Vf) and used in calculating the swelling index. The content of the measuring cylinder after 24 hours was filtered with the aid of a calico cloth. The water was completely drained into a dry measuring cylinder (10 mL). The volume of water drained from the pectin was recorded, and the difference between the initial volume of pectin mucilage and the volume of water drained was recorded as the water absorbed by the pectin. The pH, moisture content, and acid insoluble ash (AIA) of the extracted pectins were also determined using Pharmacopeia methods [19].

#### 2.2.3. Elemental Analysis

Elemental content analysis was carried out on the extracted pectin using the methods described by [20, 21]. All determinations were carried out in triplicates. Pectins from the various genotypes were dry digested, and after centrifugation, the clear supernatant digests were used for elemental analysis. The presence and amounts of iron (Fe), copper (Cu), zinc (Zn), manganese (Mn), cadmium (Cd), lead (Pb), mercury (Hg), and arsenic (Ar) in each digest were determined with an atomic absorption spectrophotometer (Buck Scientific Model 210V GP) using a hollow lamp with an appropriate wavelength (Fe, 248.3 nm; Cu, 324.8 nm; Zn, 213.9 nm; Mn, 279.5 nm; Cd, 228.9 nm; Pb, 283.3; Hg, 253.7 nm; and Ar, 193.7 nm).

The article "Utilization of Pectin from Okra as Binding Agent in Immediate Release Tablets" was published in 2021. Journal: Biomed Res Int.

#### 2.2.4. Drug-Excipient Compatibility Studies

A Bruker alpha II spectrophotometer was used to assess the compatibility of paracetamol and pectin from the different genotypes. The spectra of paracetamol, individual pectin, and physical mixtures of paracetamol and pectin were recorded by scanning in the wavelength region of 4000–400 cm^−1^ using the Bruker alpha II spectrophotometer. The spectra of the three samples were subsequently superimposed to assess if the main absorption bands present in the drug and pectin are still evident in the physical mixtures.

#### 2.2.5. Preparation of Tablets

The wet granulation method was used in formulating eighteen (18) different batches of granules as described by [18]. All ingredients (except talc) were mixed thoroughly, and a sufficient volume of ~35 ml of 10%, 15%, and 20%w/v of mucilage of the binder (pectin/tragacanth) was added gradually to the powder blend, and kneading was performed for ~20 min until formation of a dough mass with enough cohesiveness. The actual amounts of the ingredients used are depicted in Table 1(binders at 10%w/v (F1-F5), binders at 15%w/v (F7-F11), and binders at 20%w/v (F13-F17)). Prior to compression of the granules, the compressibility indices and the Hausner's ratios were determined [2]. All batches of granules were compressed into tablets with a constant compaction pressure (~120 Mpa) using a Saimach (11/37) tableting machine after talc had been incorporated into the granules.

In each formulation, the active pharmaceutical ingredient (API) was paracetamol (500 mg). Pectin from the different genotypes (PC1-PC5) was present in batches F1-F5. Pectin from the different genotypes (PC1-PC5) was present in batches F7-F11. Pectin from the different genotypes (PC1-PC5) was present in batches F13-F17. A natural polymer (tragacanth) was used as the standard binder in batches F6, F12, and F18.

#### 2.2.6. Assessment of Tablet Properties

*(1) Uniformity of Weight Test*. In each batch of formulated paracetamol tablets, twenty tablets were randomly selected and weighed cumulatively and individually using a digital analytical balance (Metler, B634930296). The average weight of the weighted tablets was determined, and the weight of the individual tablets was deducted from the average weight to calculate the individual tablet's percentage deviation from the mean [19, 22, 23].

*(2) Uniformity of Dimensions (Thickness and Diameter) of Tablets*. The thickness and diameter of twenty (20) randomly selected tablets from each batch were determined with digital Vernier callipers (Mitutoyo, CD-8-CSX). The mean and standard deviations of the readings were taken for all the batches [19, 22, 23].

*(3) Crushing Strength and Tensile Strength*. The hardness of six (6) tablets randomly selected from each batch was determined individually by diametrically compressing the tablets using Veego hardness tester (HT-1). The hardness was read on the side scale of the tester. The average hardness was then calculated for each batch. The tensile strength (*T*_*s*_) was determined using the following equation [19, 22, 23].

(1) $$\begin{array}{c} \text{Tensile strength}=\left[\frac{2F}{\pi DT}\right], \end{array}$$

where *F* (N) is the diametrical tablet break force, *D* (cm) is the diameter of the tablet, and *T* (cm) is the thickness of the tablet.

*(4) Friability Test*. The friability test was performed using the Thermomix Friability test Apparatus (C-FT-20). A number of tablets with an average weight of 6.5 g were randomly sampled from each batch, weighed, and placed in the friabilator, which was then regulated at 25 revolutions per minute. The tablets were then subjected to one hundred (100) revolutions. Tablets were subsequently dedusted and reweighed to calculate the percentage weight loss [19, 22, 23]. The percentage friability was calculated as follows:

(2) $$\begin{array}{c} \%\text{Friability}=\left\lfloor \frac{\left(W1-W2\right)}{W1}\right\rfloor \times 100. \end{array}$$

*W*_1_ is the original weight before friability test, and *W*_2_ is the final weight after the friability test.

*(5) Disintegration Test*. Six randomly selected tablets were carefully placed in each of the six cylindrical tubes of the disintegration machine (T-TD-2). The time of disintegration was taken to be the time there was no granule left on the mesh of the basket racks. The experiment was carried out in duplicate for each batch and the mean time of disintegration for each batch determined [19, 22, 23].

*(6) Assay*. The paracetamol content of the twenty tablets in each batch was determined as described by [24]. Twenty (20) paracetamol tablets were randomly sampled and weighed accurately, and the average weight was recorded. The tablets were crushed to a fine powder, and a quantity of the powder equivalent to 0.15 g of paracetamol was accurately weighed [19]. The powder mixture was dissolved in a mobile phase (methanol 65%: 0.1% TFA in water 35%) with the aid of sonication and then made up to the 100 ml mark with the mobile phase. The solution was filtered through Whatman filter paper (No. 5) into another 100 ml volumetric flask. From the above filtrate, 1 ml was taken in a 10 ml volumetric flask and volume was made up to the mark with the mobile phase, and the solution was then filtered using sintered glass filter and loaded in the injector of an Agilent HPLC (1260 with programmable absorbance detector and Agilent Zorbax SB-Phenyl 150 mm × 3.0 mm × 3.5 *μ*m column). The sample solution (1 *μ*l) was injected at a flow rate of 1 ml/min, and the detection of eluent was carried out at 230 nm. The injection was repeated three times, and the peak area of paracetamol was recorded. The average peak area was then used to calculate the amount of drug present using the average peak area of pure paracetamol with the same concentration as a standard. The experimental procedure was repeated for the other batches.

*(7) In Vitro Dissolution Test*. *In vitro* dissolution studies were carried out using the method described by [19, 24, 25]. The Veego UDA-8D USP dissolution apparatus II (paddle apparatus) was used to conduct the dissolution test. A volume of 900 ml of phosphate buffer with a pH of 5.8 was used as the dissolution media in each of the six vessels. The temperature of the dissolution media was maintained at 37 ± 2°C. 10 ml of the dissolution media was withdrawn and filtered at different time intervals of 5, 15, 30, 45, and 60 mins. Sink condition was maintained throughout the experiment. Each sample withdrawn was filtered, and 0.50 ml of each filtrate was diluted to 50 ml with the phosphate buffer. The diluted solution was then assayed spectrophotometrically at 245 nm, using phosphate buffer (pH 5.8) in the reference cell. The amount of paracetamol released was then determined from the calibration curve (*y* = 806.29*x* − 0.0784, *R*^2^ = 0.9995). The experimental procedure was repeated for the other batches. A graph of percentage drug released against time was plotted to establish the dissolution profile of paracetamol from each batch.

The article "Utilization of Pectin from Okra as Binding Agent in Immediate Release Tablets" was published in 2021. Journal: Biomed Res Int.

### 2.3. Data Analysis

GraphPad Prism 6.00 for Windows (GraphPad Software, San Diego California, USA) was used to analyze the data. *P* ≤ 0.05 was considered significantly different at 95% confidence interval.

## 3. Results and Discussion

### 3.1. Physicochemical Properties of the Okra Pectin

#### 3.1.1. Pectin Yield, pH, and Acid Insoluble Ash

After extraction, the yields obtained were in an ascending manner of PC1<PC4<PC3<PC5<PC2. Structural disparities in the backbone of pectin from the various genotypes culminated in differences in the yield of the pectins since the same extraction protocol was used [15, 17]. The pH used in the extraction process is a plausible explanation to the observed values in Table 2. It has been reported by [8–10] that lower pH can produce higher yields of pectin; however, [15, 17] also indicated that neutral pH ranges used in pectin extraction also produce pectins with lesser susceptibility to varying pH fluctuations. Furthermore, such pH values do not cause irritation on the gastrointestinal tract's mucosal lining. The amount of earthly matter present in the extracted pectins was very low due to the correspondingly low contents of acid insoluble ash (<1%) (Table 2) [26]. The potential swelling properties and water holding capacities of pectin are good indicators of their ability to from crosslinking bridges and impart cohesive and compact properties in a powder mix for tableting. The swelling indices of the genotypes differed as a result of genetic variations (Table 2) [10, 27].

#### 3.1.2. Moisture Content, Elemental Content, and Swelling Indices of Extracted Pectins

The rate of decomposition of a natural product can be affected by its moisture content. The amount of moisture in a material may affect its flow properties and microbiological stability. High moisture content may encourage microbial growth and cause some powders to clump together forming hard aggregates [28, 29]. The moisture percentage of all genotypes was less than 20%, which was lower than pectin from other sources (Table 2) [27]. Pectin from PC1-PC5 showed low contents of toxic metals (Figure 1(b)) and micronutrients (Figure 1(a)) which were within specifications as stated by [30]. This suggests the possible nontoxicity of the okra pectins, and they could therefore be used as pharmaceutical excipients.

#### 3.1.3. Compatibility of Drug and Excipient

A spectrum of pure paracetamol produces functional groups at 3322.03 cm^−1^, 3159.39 cm^−1^ (hydroxyl group, O-H stretching) and 1561.11 cm^−1^, 1504.98 cm^−1^ (amide II band) (Figure 2(a)) [19] while pectin from all the genotypes showed the following characteristic features: stretching within the range of 3100-3600 cm^−1^ (O-H stretching), bands within the range of 3000-2700 cm^−1^ (C-H stretching), bands within the range of 1730 and 1700 cm^−1^ (*C* = 0), and bands within the range of 1600 and 1670 corresponding to COOH stretching (Figure 2(b)). The physical mixture of pectin and paracetamol in Figure 2(c) contained all the major bands of the two constituents, respectively (Figures 2(a) and 2(b)). This indicates the stability and compatibility of the pectin with the paracetamol.

### 3.2. Physicomechanical Characteristics of Tablets

#### 3.2.1. Flow Characteristics of Formulated Granules

The granules prepared exhibited good flow properties based on their Hausner ratios (1.02-1.24), Carr's indices (2.70-19.41), and angle of repose (28.10-37.08°) (Table 3). The relatively smooth granulate surface, low moisture content of granules, sufficient granulate size distribution, and spherical shapes accounted for the flow depicted by the granules [2].

The article "Utilization of Pectin from Okra as Binding Agent in Immediate Release Tablets" was published in 2021. Journal: Biomed Res Int.

#### 3.2.2. Uniformity in Weight and Dimensions of Compressed Tablets

All batches passed the uniformity of weight test which is summarized in Table 4 [19, 31, 32]. All of the formulated batches had their dimensions (diameter and thickness) within the acceptable range of ±5% (Table 4) [33, 34]. Thus, the processes carried out during the preparation of the tablets comply with good manufacturing practices. Variations in tablet diameter and thickness (>±5%) will impact the convenience of blister and plastic packaging and hence patients' acceptance in ingesting the tablet.

#### 3.2.3. Crushing Strength of Compressed Tablets

A diametric crushing force of 3 kg/F is considered to be the minimum crushing force for an immediate release tablet. All the formulated tablets had crushing forces greater than 3 kg/F, thus being able to withstand fractures optimally (Table 4) [35]. Binders are added to a tablet formulation to ensure plasticity or elasticity and increase interparticulate bonding strength in the tablet. This is done to ensure that the tablet remains intact after compression [33–35]. Generally, an increase in binder concentration results in a corresponding increase in tablet hardness due to the increase in interparticulate bonding and film forming properties [1, 31, 33]. This property was exhibited by pectin from all the genotypes when they were used as binders and confirms their suitability for use as binders (Figure 3). However, there were variations in the extent to which each genotype increases tablet hardness when their concentrations as binders are increased (Figure 4).

#### 3.2.4. Tensile Strength of Compressed Tablets

Tensile strength is a measure of the bond strength of tablets. It is a basic mechanical property of a compressed tablet which maintains the consistency of tablet strength properties even if the size of the tablet is changed [13]. The tensile strength characterizes the strength of a tablet more completely than hardness. The tensile strength of all pectins extracted was highest at 20%w/v. This confirms that increasing the concentration of the pectin as binders resulted in a corresponding increase in bond strength within the tablet. Statistical analysis on the tensile strength of tablets prepared from okra pectin in comparison with the tragacanth tablets revealed statistical differences in their tensile strength (Figure 5).

The article "Utilization of Pectin from Okra as Binding Agent in Immediate Release Tablets" was published in 2021. Journal: Biomed Res Int.

#### 3.2.5. Friability Index of Formulated Tablets

All batches passed the test for friability (%friability < 1) (Table 4) [19]. This implies that there was precise regulation of tablet weight, effective granulation process, low-level of moisture, and suitable concentration of binder. The low levels of percentage friability also indicate that the manufactured batches of paracetamol tablets can endure mechanical strain and shock during processing, shipment, and handling and ultimately suggest the suitability of incorporation of okra pectins as binders in immediate release tablets.

#### 3.2.6. Disintegration Time Profile of Formulated Tablets

The process whereby tablets spontaneously break down into smaller fragments in the presence of a solvent is described as disintegration. Increasing the concentration of binders is known to increase the hardness of tablets with a corresponding increase in disintegration time [30, 31]. This effect was also observed in immediate release tablets prepared with the various pectins as binders (Figures 3 and 6). All pectins when used as binders at 10%w/v produced tablets which passed the disintegration test (*D*_*T*_ < 15 minutes). Pectin from PC4 when used as a binder at 15%w/v (F10) produced a compact tablet which was unable to disintegrate within the stipulated 15 minutes (Figure 6 and Table 4). Pectins from PC1, PC4, PC2, and PC3 when used as binders at 20%w/v, F13, F16, F14, and F15, respectively, also produced relatively compact and hard immediate release tablets which failed the disintegration test (*D*_*T*_ > 15 minutes) (Figure 6 and Table 4). Further analysis on the disintegration time of the extracted pectins as a binder with the standard binder at corresponding concentrations using *t*-test revealed significant differences (*P* ≤ 0.05) for some genotypes (Figure 7).

#### 3.2.7. Uniformity in Drug Content of Formulated Tablets

When paracetamol is used as the active ingredient in a tablet, the amount of drug in the tablet should falls between 95% and 105% of the labelled claim [19]. All the eighteen (18) formulated batches of paracetamol tablets had their drug content falling within the allowed limit (Table 4). Thus, the drug content of all the batches is considered to be optimal, as effective release in vivo would ensure the achievement of therapeutic concentration and hence enhance the therapeutic response.

#### 3.2.8. Dissolution Profile of Formulated Tablets

All the formulated tablets complied with the dissolution limit specifications with the exception of F10, F13, F14, F15, and F16 (Figure 8). The dissolution profile of the eighteen (18) formulated paracetamol tablet batches revealed that batches which were more compact and did not disintegrate within 15 minutes also failed the dissolution test (batches F10, F13, F14, F15, and F16). Pectins from PC1, PC4, PC2, and PC3 when used as binders at 20%w/v, F13, F16, F14, and F15, respectively, produced relatively compact and hard tablets which failed the disintegration test and also the dissolution test. Hence, using these pectins as binders at concentrations above 15%w/v in immediate release tablets will not produce the desired therapeutic effects. However, they may be subsequently used as potential control-releasing agents at concentrations above 20%w/v.

The article "Utilization of Pectin from Okra as Binding Agent in Immediate Release Tablets" was published in 2021. Journal: Biomed Res Int.

## 4. Conclusion

Tablet batches produced from pectin of all okra genotypes as binders at 10 and 15%w/v passed all the quality assessment tests (except PC4 at 15%w/v) and are comparable with tragacanth BP. Pectins from PC1, PC2, PC3, and PC4 when used as binders at 20%w/v produced hard and compact tablets which failed the disintegration and dissolution tests but passed all other quality control parameters. Pectin extracted from different genotypes of okra has an influence on its utilization as a binder in immediate release tablets.

## Figures and Tables

**Figure 1:** Elemental contents of extracted pectin: (a) micronutrients and (b) toxic metals.

**Figure 2:** FTIR spectra of (a) active ingredient, (b) pectin, and the (c) blend of both.

**Figure 3:** Effect of increasing concentration of pectin on tablet hardness.

**Figure 4:** Analysis on the hardness of tablets from pectin as binders ((a–c) 10%w/v, 15%w/v, and 20%w/v, respectively) and a standard binder using *t*-test. Values are mean ± SD, *n* = 6, ^∗^*P* ≤ 0.05, ^∗∗^*P* ≤ 0.01, and ^∗∗∗^*P* ≤ 0.001.

**Figure 5:** Analysis on tensile strength of tablets from pectin as binders ((a–c) 10%w/v, 15%w/v, and 20%w/v, respectively) and a standard binder using *t*-test. Values are mean ± SD, *n* = 6, ^∗^*P* ≤ 0.05, ^∗∗^*P* ≤ 0.01, and ^∗∗∗^*P* ≤ 0.001.

**Figure 6:** Effect of increasing concentration of pectin on disintegration time.

**Figure 7:** Statistical analysis on the disintegration time of tablets from pectin as binders ((a–c) 10%w/v, 15%w/v, and 20%w/v, respectively) and a standard binder using *t*-test. Values are mean ± SD, *n* = 2, ^∗^*P* ≤ 0.05, and ^∗∗^*P* ≤ 0.01.

**Figure 8:** Dissolution profiles of formulated tablets (mean ± SD, *n* = 6).

**Table 1:** Formula for formulated batches.

Formulation code	Ingredients (per tablet)				
	Pectin (%w/v)	Tragacanth (%w/v)	Starch (mg)	Lactose (mg)	Talc (mg)
F1-F5	10	-	46.5	73.5	1.0
F6	-	10	46.5	73.5	1.0
F7-F11	15	-	46.5	73.5	1.5
F12	-	15	46.5	73.5	1.5
F13-F17	20	-	46.5	73.5	2
F18	-	20	46.5	73.5	2

The article "Utilization of Pectin from Okra as Binding Agent in Immediate Release Tablets" was published in 2021. Journal: Biomed Res Int.

**Table 2:** Properties of extracted pectin.

Parameter	Okra genotypes				
	PC1	PC2	PC3	PC4	PC5
Pectin yield (%)	6.12	18.84	11.93	7.7	13.54
pH	6.92 ± 0.010	6.74 ± 0.006	6.39 ± 0.012	6.87 ± 0.006	6.80 ± 0.010
Moisture content (%)	16.2 ± 1.20	19.7 ± 0.5	11.2 ± 2.0	16.1 ± 0.6	15.9 ± 0.00
AIA (%)	0.33 ± 0.09	0.20 ± 0.03	0.23 ± 0.01	0.37 ± 0.04	0.15 ± 0.04
Swelling index (%)	405.05 ± 0.045	555.737 ± 0.015	407.246 ± 0.009	441.666 ± 0.020	540.394 ± 0.010
Water holding capacity (10 ml)	10.00 ± 0.01	10.0 ± 0.02	9.5 ± 0.01	10.00 ± 0.01	10.00 ± 0.01

**Table 3:** Flow characteristics of granules.

Code	Hausner's ratio	Carr's index	Angle of repose
F1	1.24	19.41	37.08
F2	1.13	11.29	30.92
F3	1.15	13.55	30.31
F4	1.10	9.35	30.01
F5	1.13	12.14	30.12
F6	1.09	8.56	29.47
F7	1.15	13.2	28.10
F8	1.11	10.00	28.80
F9	1.13	10.86	28.40
F10	1.07	7.21	28.40
F11	1.02	2.70	28.90
F12	1.18	16.00	27.50
F13	1.12	10.42	31.00
F14	1.01	2.70	29.00
F15	1.12	10.39	29.83
F16	1.07	6.36	29.47
F17	1.02	2.78	29.00
F18	1.05	4.45	29.00

**Table 4:** Physicomechanical characteristics of formulated tablets.

Code	Average weight (g) *n* = 20	Tablet thickness (mm) *n* = 20	Tablet diameter *n* = 20	Hardness (kg/F) *n* = 6	% friability	Disintegration time (*D*_*T*_) (min) *n* = 2	Assay (%)	Tensile strength (N/cm^2^) *n* = 6
F1	0.634 ± 0.001	4.20 ± 0.12	13.04 ± 0.01	3.22 ± 1.30	0.008	6.19 ± 1.01	99.71 ± 0.02	0.3741 ± 0.15
F2	0.634 ± 0.001	3.69 ± 0.07	13.04 ± 0.02	3.6 ± 1.30	0.015	11.14 ± 0.87	99.08 ± 0.03	0.4761 ± 0.10
F3	0.632 ± 0.008	3.87 ± 0.05	13.03 ± 0.03	4.88 ± 0.89	0.180	7.01 ± 0.81	101.16 ± 0.13	0.6158 ± 0.10
F4	0.631 ± 0.003	3.99 ± 0.17	13.07 ± 0.01	3.74 ± 1.15	0.196	7.12 ± 0.82	100.78 ± 0.15	0.4563 ± 0.14
F5	0.633 ± 0.002	3.49 ± 0.08	13.02 ± 0.03	3.56 ± 0.73	0.110	7.14 ± 0.66	98.10 ± 0.20	0.4985 ± 0.12
F6	0.630 ± 0.001	3.82 ± 0.07	13.08 ± 0.05	4.76 ± 0.96	0.003	8.12 ± 1.23	99.98 ± 0.16	0.6062 ± 0.12
F7	0.635 ± 0.003	3.59 ± 0.08	13.07 ± 0.04	3.60 ± 0.99	0.147	11.03 ± 1.02	101.55 ± 0.13	0.4882 ± 0.13
F8	0.640 ± 0.002	3.89 ± 0.09	13.08 ± 0.03	4.60 ± 1.49	0.003	13.12 ± 0.67	99.91 ± 0.05	0.5753 ± 0.11
F9	0.645 ± 0.002	3.73 ± 0.07	13.05 ± 0.02	4.96 ± 1.23	0.046	8.33 ± 0.98	97.69 ± 0.07	0.6484 ± 0.13
F10	0.637 ± 0.002	3.79 ± 0.11	13.07 ± 0.14	7.72 ± 1.61	0.003	18.43 ± 1.4	99.72 ± 0.05	0.9917 ± 0.10
F11	0.637 ± 0.003	4.14 ± 0.13	13.06 ± 0.05	4.00 ± 1.39	0.003	7.10 ± 1.02	100.05 ± 0.09	0.4707 ± 0.14
F12	0.634 ± 0.004	3.74 ± 0.10	13.07 ± 0.01	5.12 ± 1.79	0.175	8.19 ± 1.01	98.98 ± 0.03	0.6665 ± 0.12
F13	0.621 ± 0.002	3.99 ± 0.10	13.07 ± 0.01	8.8 ± 1.22	0.510	25.43 ± 1.22	98.57 ± 0.04	1.0738 ± 0.13
F14	0.647 ± 0.002	3.63 ± 0.12	13.05 ± 0.02	7.8 ± 1.06	0.158	25.14 ± 1.03	98.20 ± 0.05	1.0477 ± 0.16
F15	0.641 ± 0.005	3.59 ± 0.12	13.07 ± 0.01	7.52 ± 1.36	0.108	19.41 ± 0.88	98.22 ± 0.03	1.0198 ± 0.13
F16	0.639 ± 0.001	3.87 ± 0.13	13.06 ± 0.02	8.94 ± 0.56	0.022	21.06 ± 0.61	99.00 ± 0.08	1.1255 ± 0.14
F17	0.639 ± 0.001	3.36 ± 0.11	13.05 ± 0.03	6.7 ± 1.08	0.003	7.12 ± 0.85	99.56 ± 0.06	0.9723 ± 0.13
F18	0.639 ± 0.001	3.80 ± 0.07	13.05 ± 0.03	6.26 ± 0.97	0.405	8.14 ± 1.02	99.71 ± 0.02	0.8033 ± 0.13

The article "Utilization of Pectin from Okra as Binding Agent in Immediate Release Tablets" was published in 2021. Journal: Biomed Res Int.

## Data Availability

The data used to support the outcomes of this investigation is provided in the paper and is also accessible upon request from the corresponding author.
